RETRACTED

# Overexpression of Bacterial *mtlD* Gene in Peanut Improves Drought Tolerance through Accumulation of Mannitol

**DOI:** 10.1155/2014/125967

**Published:** 2014-11-11

**Authors:** Tengale Dipak Bhauso, Thankappan Radhakrishnan, Abhay Kumar, Gyan Prakash Mishra, Jentilal Ramjibhai Dobaria, Kirankumar Patel, Manchikatla Venkat Rajam

**Affiliations:** ^1^Directorate of Groundnut Research, Post Box No. 5, Junagadh, Gujarat 362001, India; ^2^University of Delhi, Benito Juarez Road, New Delhi 110021, India

## Abstract

In the changing global environmental scenarios, water scarcity and recurrent drought impose huge reductions to the peanut (*Arachis hypogaea* L.) crop yield. In plants, osmotic adjustments associated with efficient free radical scavenging ability during abiotic stress are important components of stress tolerance mechanisms. Mannitol, a compatible solute, is known to scavenge hydroxyl radicals generated during various abiotic stresses, thereby conferring tolerance to water-deficit stress in many plant species. However, peanut plant is not known to synthesize mannitol. Therefore, bacterial *mtlD* gene coding for mannitol 1-phosphate dehydrogenase under the control of constitutive promoter CaMV35S was introduced and overexpressed in the peanut cv. GG 20 using *Agrobacterium tumefaciens*-mediated transformation. A total of eight independent transgenic events were confirmed at molecular level by PCR, Southern blotting, and RT-PCR. Transgenic lines had increased amount of mannitol and exhibited enhanced tolerance in response to water-deficit stress. Improved performance of the *mtlD* transgenics was indicated by excised-leaf water loss assay and relative water content under water-deficit stress. Better performance of transgenics was due to the ability of the plants to synthesize mannitol. However, regulation of *mtlD* gene expression in transgenic plants remains to be elucidated.

## 1. Introduction

Peanut (*Arachis hypogaea* L.) is one of the important grain crops widely grown in tropics and subtropics with the total production areas of 21–24 M ha [1]. Peanut is generally grown under rain-fed conditions where drought is a major constraint limiting the productivity of peanut crop. Drought frequently occurs in the semiarid areas, which accounts for about 70% of the peanut growing area [2]. One of strategies to grow peanut crop in drought-prone environment is to develop peanut varieties tolerant to water-deficit stress [3]. Conventional plant breeding for drought-tolerant varieties is laborious and time consuming and commonly yields limited successes. Genetic engineering offers great potential for the improvement of peanut varieties tolerant to water-deficit stress [4].

RETRACTED

Plants have evolved multiple mechanisms to survive drought stresses. Cellular dehydration is the common phenomenon under drought environment resulting in the loss of cell turgor [5]. In order to maintain cell turgor, plants usually accumulate low molecular weight compatible solutes [6]. In response to water deficit, there were enhanced productions of compatible solutes like polyols, amino acids, and tertiary and quaternary ammonium and sulfonium compounds. These compatible solutes play vital roles in protecting cells from cellular dehydration [6, 7]. In general, accumulation of sugars, sugar alcohols, and proline [8, 9] in response to water deficit has been reported in many plant species.

It has been reported that mannitol, a kind of compatible solutes, is induced to accumulate in algae and higher plants during water deficit [10] and can be implicated in imparting drought tolerance [8, 11]. However, peanut plant is not reported to synthesize mannitol. Mannitol is a six-carbon, noncyclic sugar-alcohol having its role in the coenzymes regulation, scavenging of free-radical, storage of energy, and osmoregulation [12]. The* mtlD* is a bacterial gene that encodes mannitol 1-phosphate dehydrogenase. Transgenic plants carrying* mtlD *convert mannitol 1-phosphate to mannitol via nonspecific phosphatases [13]. Overexpression of the genes involved in the biosynthesis of osmolytes, such as mannitol [8, 14], trehalose [15], and many more in various transgenic plants showed increased abiotic-stress tolerance.

The* mtlD* gene has been transferred to several crop species like wheat [16], eggplant [17], sorghum [18], and Maize [19] resulting in enhanced plant height, fresh and dry biomass weight, increase in salinity, and/or drought tolerance [20, 21]. In these plants, biosynthesis and accumulation of mannitol increased, while its catabolism decreased under stress conditions [3, 22].

Mannitol is used as an additive in many processed foods and its overexpression is known to be a useful tool in enhancing crop resistance to drought [23]. Therefore, introducing novel genes encoding enzymes involved in biosynthesis of compatible solutes like mannitol could be a better alternative to conventional breeding to improve peanut varieties tolerant to drought stress [24]. An approach to improve abiotic stress-tolerance by introducing* mtlD* gene into peanut genome could be promising [11, 17].

In the present study, we report the successful introduction and overexpression of* mtlD* gene cloned from* Escherichia coli* to the peanut cv. GG20, which is one of the most popular varieties of India, under the control of CaMV35S constitutive promoter. Overexpression of* mtlD* gene has resulted in the synthesis of mannitol and conferred increased tolerance of drought stress in the transgenic peanut.

RETRACTED

## 2. Materials and Methods

### 2.1. Plant Material and Culture Conditions

The seeds of peanut were surface sterilized with 70% ethanol for 1 min and 0.1% (w/v) HgCl_2_ for 3 min and rinsed three times with sterile distilled water. The testa was removed in a laminar air flow hood; embryos were removed; and excised cotyledons were used as explants. The cultures were done in modified MS medium [25] and maintained at 26 ± 1°C, 16 h photoperiod with cool white fluorescent light of 42 *μ* mol m^−2^ s^−1^ illumination for 15 d and then subcultured in medium containing 15 mg/L BAP.

### 2.2. Plasmid and Transformation Vector

The* mtlD* gene of* E. coli* which was originally isolated by Prof Hans J Bohnert (University of Illinois, USA) was used. The gene cassette had the 1149 bp coding region of* mtlD*, downstream of a CaMV35S promoter in the binary vector pCAMBIA 1380 containing a plant selectable marker gene,* npt*II (Figure 1).

### 2.3. Plant Transformation, Selection, and Regeneration of Transformed Tissues

The excised cotyledon and immature leaf explants from mature presoaked seeds were transformed with* A. tumefaciens* strain LBA4404 harboring the binary plasmid pCAMBIA1380:*mtlD* gene. The explants were infected with resuspended* A. tumefaciens* culture for 20 min at room temperature under continuous shaking and transferred on to cocultivation medium for 3 days at 26 ± 1°C [25]. After transformation, the explants were rinsed 5-6 times with sterile water followed by a wash with cephataxime (Lupin, India) (200 mg/L), blotted to remove excess bacterial suspension, and cultured in the shoot inducing medium. To eliminate overgrowth of* A. tumefaciens*, the medium was also supplemented with cephataxime (Lupin, India) (200 mg/L).

The 1-2 cm long healthy shoots were transferred to MS basal media without hormones and grown for a week, before transferring to rooting medium. The shoots that survived the kanamycin selection were rooted on MS medium supplemented with 1 mg L^−1^ NAA, 250 mg L^−1^ cefotaxime, and 100 mg L^−1^ kanamycin. The explants were subcultured at 15 d interval. The plantlets with well-developed roots were transferred to earthen pots for hardening and hardened plants were grown in a PII containment facility. The explants without Agrobacterium-infection were used as negative control.

### 2.4. Molecular Confirmation of Putative Transgenic Plants

PCR-analysis was done on the putative transgenics using gene-specific primers to pick up transgenics carrying the* mtlD* and* npt*II genes [26]. Genomic DNA was extracted from the young leaves of kanamycin-resistant and wild-type (WT) plants using the DNAzol kit (Molecular Research Center, Inc.). The plasmid DNA was also amplified with respective primers as positive control. The PCR reaction (20 *μ*L) is comprised of 2 *μ*L 10x PCR buffer (Fermentas), 1 *μ*L genomic DNA (100 ng), 1.6 *μ*L dNTP mix (2 mM), 1 *μ*L forward and reverse primers (25 pM each), and 1 U* Taq* DNA polymerase (Fermentas).

RETRACTED

The pair of primers for the detection of the* mtl*D coding region is* mtl*D-Fwd: 5′-GGGCAGGTGAAACGTAAAGA-3′ and* mtl*D-Rev: 5′-CAGTTTACGCAGTGGCTGAC-3′ (annealing temperature 60°C; product size 600 bp) and, for the* npt*II gene,* npt*II-Fwd: 5′-GAGGCTATTCGGCTATGACTG-3′ and* npt*II-Rev: 5′-ATCGGGAGCGGCGATACGTA-3′ (annealing temperature 56°C; product size 750 bp).

PCR reactions were set up with the following thermal profile: 94°C for 4 min, followed by 35 cycles of 94°C for 1 min, 60°C or 56°C (for* mtl*D and* npt*II, resp.) for 45 s, and 72°C for 1 min and final extension at 72°C for 7 min. The amplified product was resolved on 1.2% agarose gel, visualized by Ethidium bromide staining, and documented using a Fuji FLA5200 imaging system.

### 2.5. RNA Isolation and RT-PCR

Total mRNA was isolated from eight lines obtained from independent transformation events (MTD1-8 in T_2_ generation) and the WT using RNA extraction kit (Qiagen) and subjected to RNase-free DNase I (Fermentas) digestion and purification [26]. The RNA was quantified using ND-1000 spectrophotometer (NanoDrop Technologies Inc., USA). Equal amount of RNA from each sample was used for the two-step RT-PCR reaction. The first-strand of cDNA was synthesized from 1 *μ*g RNA per sample using first strand cDNA synthesis kit (Fermentas) and the product obtained was further used for second-strand amplification using gene specific primers via PCR.

### 2.6. Segregation Analysis

Selected T_0_ plants with sufficient number of seeds were selected for segregation analysis [26]. The T_1_ progeny of the five lines was grown in pots under controlled conditions in a PII containment facility. The plantlets at 2–4-leaf stage were used for PCR analysis using gene-specific primers to score the amplicons. The *χ* ^2^ test was conducted in the progenies from all the events on the basis of expected and observed frequencies.

### 2.7. Southern Blot Analysis

Genomic DNA (30 *μ*g) of transgenic and WT plants was individually digested with* EcoRI*, separated on 0.8% agarose gel, and then transferred to Biodyne plus (0.45 *μ*m) nylon membrane (PALL Life Sciences) using alkaline transfer buffer (0.4 N NaOH and 1 M NaCl). The* mtlD* probe (285-bp), labelled with thermostable alkaline phosphatase, using alkaphos direct labelling kit (Amersham, GE Healthcare, UK), was used for hybridization. Hybridization was carried out overnight at 55°C in hybridization buffer (Amersham, GE Healthcare, UK) and membrane was washed (at 55°C for 15 min) first in primary wash buffer (25 mL) and then in secondary wash buffer at room temperature. Hybridized membrane was detected by using CDP-star chemiluminescent as substrate and signals were visualised on Amersham Hyperfilm ECL after 1 h.

RETRACTED

## 3. Water Stress Experiments

The 45 d old* mtlD* transgenic plants in T_2_ generation and WT lines which were grown under PII containment facility were used for water-deficit stress tolerance studies after withholding the irrigation for 24 days. All the eight independent transgenic lines, namely, MTD1-8 along with WT, were evaluated for the following parameters.

### 3.1. Estimation of Mannitol Level

Mannitol was extracted from the leaves (WT and T_2_ transgenic) and quantified by binary gradient High Performance Liquid Chromatography (Shimadzu LC 10 series) as described by Tarczynski et al. [14]. For separation, 10 *μ*L sample was injected per run (operated at 1 mL min^−1^) with acetonitrile: water (80 : 20) as mobile phase using 5 *μ* Luna, NH_2_ 100 Å column (at 40°C) and RI detector was used for detection. Mannitol (SRL; 10 mg L^−1^) was used to develop the calibration curve to optimize the mannitol separation by diluting it to four concentration levels of 1 mg L^−1^, 2 mg L^−1^, 5 mg L^−1^, and 10 mg L^−1^. The concentration value is calculated from the area/height of the peaks on the calibration curve [8].

### 3.2. Excised-Leaf Water Loss Assay

The assay as proposed by Pierce and Raschke [27] was used with minor modification. First fully expanded leaves on the main stem from transgenic and WT plants (03 leaves each) grown under well watered conditions were excised early in the morning and placed in abaxial side up in open petri dishes. The leaves were then exposed to a light intensity of 538 *μ* mol m^−2 ^s^−1^ (incandescent) for 8 h in a growth chamber. The loss in weight was recorded for 8 h at 60 min interval. After incubation, the percentage loss in fresh weight over the unincubated control was calculated.

### 3.3. Relative Water Content (RWC)

The fresh leaf discs were used to measure RWC as per Barrs and Weatherley [28]. Initial fresh weights (FW) were measured prior to floating in petri-plates containing water (8 h) for hydration and were weighed again to measure the turgid weight (TW). It is then dried in a hot air oven (80°C for 72 h) and weighed till a consistent dry weight (DW) was obtained. RWC was calculated as RWC = [(FW − DW)/(TW − DW)] × 100.

RETRACTED

### 3.4. Statistical Analysis

The experiments on mannitol content, excised-leaf water loss assay, and RWC were set up in completely randomized design (CRD) in three replications. The significance of the treatment effects was determined by one-way ANOVA of SPSS 11.0 (Statistical Package For Social Sciences, SPSS Inc., Illinois) at 5% probability level using Tukey test. The goodness of fit of the observed segregation ratio for the* mtlD* transgene in T_1_ generation was tested against the Mendelian segregation ratio (3 : 1) using the chi-square (*χ* ^2^) test.

## 4. Results

### 4.1. Tissue Culture and Transformation

*In vitro* regeneration from the excised cotyledons of peanut resulted in direct shoot initiation after 100–105 d. Transformation efficiency was evaluated as the number of independent transgenic lines with respect to the initial number of explants cultured. In the present investigation, 1096 explants, which are cultured in 15 batches, could produce 865 shoots. After 6 weeks of culture on the selection medium, 532 (61%) shoots survived in selection medium of which 193 (45%) shoots survived under PII containment facility (Figures 2(a) to 2(g)). Finally, only 10 shoots (5.18%) were found to be PCR positive when screened with transgene specific primers (Table 1). Though the regeneration frequency recorded was quite high, the number of confirmed independent transgenic events finally obtained was relatively low. Similar trend has been observed by Kumar et al. [29] and Tiwari et al. [30]. All transgenic lines appeared normal in morphology and development.

### 4.2. Integration of Transgene in Host Genome

Kanamycin-resistant T_0_ transgenic plants were subjected to PCR analysis using transgene specific primers so as to confirm the integration of the transgenes, namely,* mtlD* and* npt*II. PCR analysis detected the presence of 600 bp amplicon of the* mtlD* and 750 bp of* npt*II (Figures 3(a) and 3(b)) genes, confirming the presence of the transgenes. Southern hybridization was also carried out with T_0_ transgenic plants to check the integration and copy number of the transgene in putative transgenic plants. All the putative transgenic plants tested positive having single copy number of transgene, while the untransformed plant tested negative (Figure 3(c)).

### 4.3. Expression of the Transgene

RT-PCR analysis was performed on the PCR positive plants to confirm the expression of the* mtlD* transcript in transgenic (T_0_) plants. 18S rRNA was used as an internal reference to normalize the initial cDNA content among samples. The result showed that the transgenic lines have expressed the* mtlD* gene at transcript level whereas no amplification was observed in untransformed plants (Figure 3(d)). There were some differences in the intensity of the RT-PCR bands. The transgenic lines MTD1, 2, and 8 showed higher mRNA titers in comparison to other lines.

RETRACTED

### 4.4. Segregation Analysis

All the selected eight T_0_ plants were found fertile and produced seeds. The progenies of these* mtlD* positive transgenics were further tested for the segregation by chi-square analysis. The segregation pattern for* mtlD* gene in T_1_ plants showed a 3 : 1 ratio, expected for single dominant gene inheritance, for six out of eight transformed lines studied (Table 2). Similar segregation pattern of transgene was also reported by Cheng et al. [31] and Tiwari et al. [30].

### 4.5. Characterization of Transgenic Peanut

#### 4.5.1. Accumulation of Mannitol

All the transgenic lines expressed* mtlD* transgene under PII containment facility. Mannitol content recorded under well-watered and water-deficit stress condition in transgenic lines ranged from 1.81–2.98 *μ*g g^−1^ to 3.02–4.74 *μ*g g^−1^ FW of tissue, respectively (Table 3). Under water-deficit stress, different transgenic lines had significantly different levels of mannitol suggesting multiple mechanisms controlling the activity of the enzyme encoded by the transgene and the level of gene expression [32].

#### 4.5.2. Excised-Leaf Water Loss Assay

After 4 h under dehydration conditions, the detached leaves of the* mtlD* overexpressing peanut plants lost less water than the detached leaves of the WT plants (Figures 4 and 5). This may be due to the greater mannitol accumulation in transgenic plants than in WT.

#### 4.5.3. Relative Water Content (RWC)

Under both well-watered and water-deficit stress, all the transgenics had significantly higher RWC over WT. Transgenics exhibited less reduction in the RWC than WT under water-deficit stress which was indicative of greater tolerance for water-deficit stress (Figure 6).

## 5. Discussion

Mannitol accumulation in* mtlD* transgenics is expected to confer a range of biotic and abiotic-stress tolerance [8, 11, 33]. Although mannitol is synthesized in various plant species, it is absent in peanut. Under stress, 1.31- to 1.82-fold increase in mannitol content was observed in different transgenics compared to the nonstressed transgenics (Table 3). When compared to the nonstressed plants, 3–10 folds of mannitol accumulation in transgenics egg plants have been reported by Prabhavathi et al. [17]. An increased accumulation of mannitol in the transgenic peanut lines indicates their tolerance capacity against drought-stress [33].

In earlier reports, transgenics with different levels of mannitol in their tissues have been shown to be tolerant to different type of abiotic stresses [3, 11]. The results of Nagabhyru et al. [34] also suggest that an endophytic fungus* Neotyphodium coenophialum* assists in imparting drought tolerance in tall fescue, by the accumulation of many compatible solutes like proline and mannitol. This supports that the level of mannitol accumulated in the tissues may act as osmoprotectant and protect the cells from free radicals and, in addition, induces several stress tolerance pathways which result in increase in their abiotic stress tolerance ability [8, 12, 18, 35].

RETRACTED

The dynamic loss in fresh weight of excised leaves by desiccation was used as a quick and convenient method of estimating the degree of water stress [36, 37]. Differences in the capacity to conserve water in different transgenic lines were observed when drought stress was imposed on transgenics. Transgenic line MTD8 presented higher capacity to conserve their water over other transgenic lines (Figures 4 and 5). Under well-watered conditions, however, no significant differences were observed in capacity to conserve their water among these genotypes. Similar results were recorded by other workers for different transgenics when evaluated using excised-leaf water loss assay [36, 37].

RWC is a physiological index related to the uptake of water by the roots, water loss by transpiration, and closure of stomata. We measured the leaf RWC since it is considered a suitable indicator for plant tissue water retention capacity and acts as an appropriate parameter to measure water status and osmotic adjustments of plants under abiotic stresses [11, 38]. Also, when the leaf RWC is reduced below some critical threshold (e.g., below 0.3 g H_2_O g^−1^ DW), there is insufficient water for preferential hydrations [39]. Transgenics peanut expressing* mtlD* gene displayed less reduction in the RWC than WT under water-deficit stress (Figure 6), supporting the reports of Karakas et al. [20] in tobacco, Abebe et al. [3] in wheat, Hema et al. [35] in finger millet, and Rai et al. [38] in tomato indicating that transgenics plants could effectively retain more water-content under drought-stress, with minimum reduction in RWC.

The present results agree with Nguyen et al. [19] work in transgenic maize where* HVA1* and* mtlD* genes resulted in improved total biomass and showed greater water use efficiency under drought conditions. The exact mechanism of* mtlD* induced regulation, responsible for improved physiobiochemical and growth-parameters under various stresses, is yet to be deciphered. Further analysis is required to study the expression pattern of* mtlD* gene when used with stress inducible promoter for the creation of transgenic peanut.

RETRACTED

In the era of global warming, drought can be a devastating problem, leaving peanut farmers with very low yields and less farm incomes. Our results established that the overexpression of* mtlD* using transgenic approach confers water-deficit stress tolerance in peanut crop by way of accumulating the mannitol. In addition to acting as an osmoregulator, sugar alcohols also maintain the enzyme-activity in a cell by maintaining the surface bound water of protein and keeping its conformation in solution [40] and displayed antioxidant activities [41] leading to increased tolerance to water deficit stress in transgenic peanut.

Although, many transgenic peanut lines have been developed across the world by different group of researchers with various degrees of improved abiotic stress tolerance but, till-date, no commercial varieties are released [42, 43]. Therefore, multiyear, multilocation field testing of the developed transgenic lines is required to further confirm the drought tolerance under actual field conditions [19]. Subsequently, the* mtlD* transgenic peanut lines, when released, are expected to improve farmer's profits in the regions of the world where unexpected and recurrent drought is one of the main factors limiting the peanut productivity. Besides, it can also be utilized as valuable prebreeding resource in the peanut improvement programme on abiotic stresses.

## Figures and Tables

**Figure 1:** Schematic representation of the T-DNA region of pCAMBIA 1380 binary plasmid used for transformation of deembryonated cotyledons with* Agrobacterium tumefaciens* strain LBA 4404. The position of the primers used in PCR assays is shown by arrows on top of the* mtlD* gene. LB, left T-DNA border sequence; RB, right border sequence; 35S, CaMV35S promoter; and* mtlD*, mannitol-1-phosphate dehydrogenase.

**Figure 2:** Genetic transformation and regeneration of peanut from deembryonated cotyledons. (a)-(b) Deembryonated cotyledons cocultured with* Agrobacterium* strain LBA4404; (c) shoot buds initiating from cocultured deembryonated cotyledons; (d) sequential regeneration process of shoots from deembryonated cotyledon explant in various concentration media; (e) transformed (green) and nontransformed shoots (yellow) in Kanamycin selection media; (f) transformed healthy shoots in Kanamycin selection media containing NAA; and (g) transformed groundnut plant with well-developed shoots transferred in pots for hardening.

**Figure 3:** Molecular characterization of* mtlD* peanut transformants. (a) PCR amplification using* mtlD* gene-specific primers (expected size 600 bp); (b) PCR amplification of transformants using* npt*II gene specific primers (expected size 750 bp), where lane N: negative control; lane P: positive control (pCAMBIA1380 plasmid DNA); and lanes 1–8: transgenic lines (MTD1 to MTD8); (c) Southern blot analysis of transgenic (T_0_) and nontransformed peanut lines. Where lanes 1–4: DNA from transgenic lines, lane 5: DNA from nontransformed line (cv. GG 20, −ve control), and lane 6: plasmid DNA (+ve control); (d) detection of* mtlD* gene transcription in transgenic plants using RT-PCR. Lane N = nontransformed line; lanes 1–8 = transgenic lines (MTD1 to MTD8), bottom row: 18SrRNA as internal control.

RETRACTED

**Figure 4:** Representative picture of excised-leaf water loss assay where detached leaves of transgenic (T) plants showed less water loss in a given time-span over wild-type (WT) plants.

**Figure 5:** Excised-leaves water loss assay shows significantly higher water loss in WT whereas reduced water-loss was found in* mtlD* transgenics. Data are average ± SE from three independent experiments; bars on the top represent the LSD_0.05_. Bars having same lower-case letters within treatments are not significantly different (*P* ≤ 0.05).

**Figure 6:** Effect of imposing water-deficit stress at full-growth stage in transgenic lines (MTDs) and WT (GG 20) on RWC content. Values are mean of three replicates and bars indicate ±SE; bars on the top represent the LSD_0.05_. Bars having same lower-case letters within treatments are not significantly different (*P* ≤ 0.05).

**Table 1:** Genetic transformation and regeneration of peanut explants from the cultivar GG 20.

Number of cocultivations	Total explants cocultured	Shoots produced	Shoots passed antibiotic selection	Shoots produced roots	Plantlets hardened and survived in glasshouse	Final recovery of putative transgenics
15	1096	865	532 (61)^*^	431 (81)	193 (45)	10 (5.18)

^*^Values in parenthesis are percentage.

**Table 2:** Segregation analysis of defensin gene in selfed progenies (T_1_) derived from *mtl*D transgenic peanut plants.

Transformed groundnut lines	Number of plants			Observed ratio	Test ratio	*χ* ^2^	*P* value
	Total	*mtlD+ *	*mtlD− *				
MTD1	54	41	13	3.15 : 1	3 : 1	0.025	0.8744
MTD2	79	59	20	2.95 : 1	3 : 1	0.004	0.9482
MTD3	82	62	20	3.1 : 1	3 : 1	0.016	0.8993
MTD4	31	22	9	2.44 : 1	3 : 1	0.269	0.6041
MTD5	16	10	6	1.66 : 1	3 : 1	1.333	0.2482
MTD6	10	7	3	2.33 : 1	3 : 1	0.133	0.7153
MTD7	20	15	5	3 : 1	3 : 1	0.000	1.000
MTD8	24	16	8	2 : 1	3 : 1	0.889	0.3457

*P* = 0.05, df = 1.

**Table 3:** Effect of imposing water-deficit stress on 45-day-old plants (T and WT) after 24 days of stress imposition on mannitol content.

Line No.	Mannitol content (*μ*g/g FW)	
	Water-deficit stress	Well watered
MTD1	3.02 ± 0.31^d^ ^z^	2.25 ± 0.29^ab^
MTD2	3.30 ± 0.42^cd^	1.81 ± 0.22^b^
MTD3	4.74 ± 0.41^a^	2.98 ± 0.38^a^
MTD4	3.72 ± 0.10^bcd^	2.83 ± 0.16^a^
MTD5	4.65 ± 0.33^a^	2.74 ± 0.29^a^
MTD6	4.26 ± 0.22^ab^	2.84 ± 0.14^a^
MTD7	3.58 ± 0.17^bc^	2.71 ± 0.29^a^
MTD8	4.12 ± 0.39^abc^	2.73 ± 0.29^a^
GG 20 (WT)	ND	ND

LSD	0.90	0.80

The data are mean of three replicates ± SE; ND: not detected; ^z^means followed by the same lower case letters within a column are not significantly different (*P* ≤ 0.05).
